# Nestin Regulates Keap1-Nrf2-HO-1-Mediated Antioxidant Responses during Stress and Malignant Hematopoiesis

This article has been retracted.

**DOI:** 10.1155/2022/1706585

**Published:** 2022-05-28

**Authors:** Chunjuan Lu, Jin Wei

**Affiliations:** ^1^Department of Blood Transfusion, Heilongjiang Provincial Hospital, Harbin, Heilongjiang 150036, China; ^2^Department of Nutrition, Heilongjiang Provincial Hospital, Harbin, Heilongjiang 150036, China

## Abstract

**Objective:**

To investigate the role of nestin in regulating Keap1-nuclear factor erythroid-2-related factor 2 (Nrf2)-heme oxygenase-1-(HO-1-) mediated antioxidant responses in stress and malignant hematopoiesis.

**Methods:**

The mRNA of peripheral blood mononuclear cells was extracted from 20 leukemia patients and 20 healthy people who were hospitalized in the Hematology Department of our hospital from September 2020 to December 2021, and the mRNA levels of nestin, Keap1, Nrf2, and HO-1 were detected by real-time- (RT-) PCR.

**Results:**

Compared with healthy controls, the mRNA of nestin, Keap1, Nrf2, and HO-1 in peripheral blood mononuclear cells of leukemia patients was significantly upregulated.

**Conclusion:**

The occurrence and development of leukemia are closely related to nestin regulating Keap1-Nrf2-Ho-1 signal pathway. *Research Significance*. This study determined the effect of nestin on the biological behavior of leukemia cells and its possible mechanism and confirmed that nestin may be a marker of tumor and tumor blood vessels.

## 1. Introduction

Leukemia is recognized as one of the major malignant tumors threatening the health of Chinese residents. Abnormal leukemia hematopoietic stem/progenitor cell proliferation and apoptosis of a group of highly heterogeneous cloned blood malignancies, formed by the leukemia cells, have unlimited proliferation ability but lose the ability of further matured and stagnation in the different phases of the cell development, unable to form mature blood cells, and normal hematopoiesis is restrained [1, 2]. Leukemic cells proliferate and accumulate in bone marrow and other hematopoietic tissues and infiltrate into other tissues and organs, resulting in a series of clinical manifestations with fever, bleeding, and anemia as the main symptoms. Lymphoblastic leukemia and myelocytic leukemia are classified according to their cell types. According to the course of disease and the degree of differentiation of leukemia cells, it is classified into acute myelocytic leukemia and chronic leukemia. It is reported that the incidence of leukemia in China is about 5.17/100,000, accounting for 1.94 of all tumors, which is the 13th place, and the ratio of male to female patients is 1.29 : 1. The death rate of leukemia was 3.94 per 100,000 people, accounting for 2.29 percent of all cancer patients, ranking ninth. This shows the develop leukemia research to have important significance [3–5].

Leukemia is a malignant hematopoietic tumor that results from abnormal hematopoietic cells. Leukemia cells are malignant cells derived from normal blood cells. In 2011, Douglas Hanahan and Robert A. Weinberg wrote Hallmarks of Cancer: Review of The Next Generation [6], elucidating 10 basic characteristics of tumor cells, namely, tumor cells mainly include the following ten characteristics: self-sufficiency of growth signals, antigrowth signal is not sensitive, resistant to cell death, the potential ability of replication, persistent angiogenesis, invasion and metastasis, avoid inflammation, immune to destroy, and promote tumor cell energy anomalies and genomic instability and mutation [7]. Leukemia cells have the basic characteristics of malignant tumor cells mentioned above, and their biological behaviors are mainly characterized by malignant proliferation, blocked apoptosis, and differentiation disorders [8].

Current studies have proved that nestin may be a marker of tumors and tumor blood vessels [9, 10]. In recent years, nestin has also been reported to be expressed in leukemia. Studies have shown that nestin protein is expressed in bone marrow smears of AML and ALL patients to varying degrees, but there is no correlation between nestin expression and patient prognosis [11]. Currently, there are few studies on the mechanism of nestin in leukemia. It has been reported that in AML models, the maintenance of HSC homeostasis depends on nestin +MSC cells, while leukemia cells destroy nestin +MSC cells [12]. However, in the ALL mouse model, nestin protein is involved in the formation of drug-resistant niche, which plays an important role in protecting leukemia proliferating cells [13]. Currently, it has been found that nestin is expressed in leukemia, but there are few studies on the role of nestin in leukemia. Therefore, this experiment is aimed at exploring the effect of nestin on the biological behavior of leukemia cells and its possible mechanism of action.

## 2. Methods

### 2.1. Participants

This study was approved by the ethics Committee of our hospital and informed consent of patients. The peripheral blood mononuclear cells (MNCS) used to detect nestin mRNA were collected from 20 patients admitted to the Hematology Department of our hospital from September 2020 to December 2021 and diagnosed with myeloid leukemia. Bone marrow cell morphology and histochemical staining were performed on all patients for FAB typing. At the same time, 20 healthy people in our hospital were collected as control.

### 2.2. Treatment of Peripheral Blood Samples

They went to the hematology department of our hospital, and after obtaining the consent of the hematology doctor, 1 ml peripheral blood was taken into the EP tube. Record the patient's hospitalization number, name, diagnosis, and number; after returning to our laboratory, the peripheral blood samples were taken out, and 1 ml normal saline was slowly added along the wall of EP tube and gently mixed to prevent RBC fragmentation; 2 ml of lymphocyte separation solution was placed in the centrifuge tube. Peripheral blood was added slowly along the wall of the centrifugal tube. The centrifuge tube was put into a centrifuge and centrifuged at 2500 r/min at 20°C for 5 min. After centrifugation, the liquid surface was divided into four layers, including plasma layer, white blood cell layer, lymphocyte separator layer, and red blood cell layer from top to bottom. The white blood cell layer was carefully sucked into an EP tube with a pipette and centrifuged at 4°C at 1000 r/min for 5 min. The supernatant was removed, and the white blood cells were cleaned once with LML normal saline and centrifuged at 4°C 1000 r/min for 5 min. Remove normal saline, add 1 ml TRIzol, carefully blow away the bottom cell masses, and store at -80°C.

### 2.3. The Expression of Nestin and Related Genes in Peripheral Blood Mononuclear Cells of Patients with Leukemia Was Detected by RT-PCR

MRNA was extracted by TRIzol and quantified by NanoDrop 2000 ultra-micro spectrophotometer. cDNA reverse transcription and fluorescence real-time quantitative reaction of mRNA were performed according to the instructions. Take GADPH as internal reference and use the formula of 2^-△△Ct^ to calculate.

### 2.4. Data Statistics

The experimental data were expressed as *X* ± *S*. SPSS 17.0 software was used for statistical analysis. Homogeneity of variance test and one way ANOVA was used for comparison between groups. SNK test (Student-Newman-Keuls method) was used for further pair comparison between groups if the variances were uniform. If variance is not uniform, Games-Howell test is used. *P* < 0.05 was considered as statistically significant difference.

## 3. Results

### 3.1. General Patient Information

Among the 20 patients with myeloid leukemia, there were 12 males and 8 females, including 15 patients with acute myeloid leukemia and 5 patients with chronic myeloid leukemia. See Table 1 for relevant information.

### 3.2. The Expression of Nestin mRNA in the Myeloid Leukemia Group and Control Group

Compared with the control group, the expression of nestin in patients with myeloid leukemia was significantly higher in Figure 1 (*P* < 0.05).

### 3.3. The Expression of Keap1, Nrf2, and HO-1 mRNA in the Myeloid Leukemia Group and Control Group

Compared with the control group, the expression of Keap1, Nrf2, and HO-1 in patients with myeloid leukemia was significantly higher in Figure 2(*P* < 0.05).

## 4. Discussion

Nestin protein is a class VI intermediate filament protein. In 1985, Hockfield and McKay first found nestin protein in embryonic rat neural tube cells [14]. Nestin positive cells decreased rapidly with embryonic maturation. When rat neural precursor cells completed migration and differentiation [15], nestin protein gradually stopped expression; so, nestin protein is considered to be a marker of neural precursor cells. Nestin gene structure is similar to class III and class *n* intermediate silk proteins [16], but nestin protein intron arrangement order, C-terminal and N-terminal amino acid number and arrangement order, and intracellular distribution position are significantly different from other five types of intermediate silk proteins; so, it is named class VI intermediate silk proteins [17, 18]. The rat nestin gene contains five exons and four introns. The first and second introns are enhancers, which activate [LA] O nestin protein during the development of midbrain and central nervous system, respectively. The molecular weight of nestin protein is 240 KD, and the C end contains 1479 amino acids and participates in the formation of heterodimers with vimentin [19], desmin [20], and interniexin [21]. Nestin protein was first known as a marker of neural stem cells. When neural embryos were formed, neural plate skin cells began to express nestin protein. When neural stem cells migrated gradually, the expression of nestin protein gradually decreased, and a-interniexin and vimentin began to express and form an intermediate filament network. In addition, nestin protein has also been found in other tissues and cells or in the process of tissue formation, such as pancreatic and liver cells during embryogenesis, but it is only expressed in immature cells. When the cells mature, nestin protein stops expressing. When the cell is mature, it will be reexpressed in the tissue [22].

Leukemia is a group of highly heterogeneous hematological tumors with malignant proliferation, blocked apoptosis, and impaired differentiation of hematopoietic cells. At present, the etiology and pathogenesis of leukemia are not very clear, and it is still an incurable disease. Gene abnormality is one of the “killers” of malignant biological behavior of leukemia cells [23–25]. Studies have shown that nestin is related to the degree of malignancy, metastasis, poor prognosis, and drug resistance of some tumors [23, 26–28], but there are still very few studies in leukemia, and it is unclear whether nestin is related to leukemia. Therefore, it is of great significance to explore the expression and function of nestin in leukemia. In view of this, the expression and role of nestin in leukemia is not very clear. Hence, this study detected the expression of nestin in leukemia patients at the mRNA level, which has clinical significance.

The abnormal antioxidant capacity of tumor is considered to be one of the mechanisms of its malignant progression. Nrf2 is a key transcription factor regulating cell redox balance. The enhancement of antioxidant capacity caused by its abnormal activation is an important reason for tumor drug resistance. Systematic analysis of the molecular mechanism of Nrf2 signaling pathway regulating oxidative stress in tumor cells is of great significance to reveal the occurrence and development of tumor and chemotherapy resistance. Studies have shown that intermediate filament protein, as a member of cytoskeleton, helps cells resist various external stresses, especially oxidative stress, and plays a cytoprotective role. Studies have shown that the expression of nestin in tumor cells is abnormally increased, which is closely related to the level of intracellular ROS, mitochondrial morphological work (oncogene. 2016), and cell aging (NAT common. 2018). However, how to regulate the redox mechanism of tumor cells and its biological significance in the progression of malignant tumors needs to be clarified. At the same time, some studies have revealed that nestin can inhibit the ubiquitination proteasome degradation of Nrf2 by Keap1 through competitive binding to Keap1 and promote the oxidative stress ability and chemotherapy resistance of lung cancer. Therefore, this study explores the relationship between nestin and Keap1 and Nrf2 [29].

Nrf2 gene deletion will reduce the hematopoietic reconstitution ability after hematopoietic stem cell transplantation, which indicates that Nrf2 is a key factor to maintain the characteristics of hematopoietic stem cells. The Keap1-nrf2 system is involved in the differentiation of hematopoietic stem cells and the maintenance of stem cell characteristics [30]. Recently, we found that the activation of Nrf2 promotes the differentiation of hematopoietic stem cells, which is conducive to the renewal of granulocytes or monocytes, while erythrocytes and lymphocytes are compensated. Therefore, the activation of Nrf2 inhibits the differentiation of hematopoietic stem cells into erythroid and lymphoid systems and promotes their transformation into granulocytes. The effect of Nrf2 on hematopoietic differentiation exists not only in normal hematopoietic stem cells but also in cells of acute myeloid leukemia [31]. Nrf2 activation promotes the expression of vitamin D receptor and RXR by activating AP-1 (activator protein-1) and promotes the cell differentiation of acute myeloid leukemia caused by 1,25-vitamin D3. This also makes it possible to inhibit Nrf2 gene as a strategy for leukemia differentiation therapy [32–34]. HO-1 is the downstream factor of Nrf2. Therefore, HO-1 changes with the change of Nrf2. Therefore, Keap/Nrf2/HO-1 is closely related to the treatment of leukemia. Our results show that leukemia is affected by nestin regulated Keap/Nrf2/HO-1 signaling pathway.

The number of cases included in this study is too small, and there are certain limitations for the classification analysis of leukemia types. We will conduct verification in more leukemia patients with different types in the subsequent study.

## 5. Conclusion

Nestin protein belongs to class I intermediate filament protein, which is involved in the construction of cytoskeleton and is mainly expressed in cells with low differentiation. It is reported that nestin protein is not only involved in the differentiation and proliferation of normal cells but also expressed in a variety of tumor cells, and participates in multiple cellular pathways related to tumor cell proliferation. In leukemia, nestin protein may regulate oxidative stress pathways such as Keap/Nrf2/HO-1, which provides a new direction for the study of leukemia formation mechanism and treatment of leukemia. Nestin protein as a marker of neural stem cells, its expression in tumor cells, redefines its identity, but the role of nestin protein in leukemia still needs a lot of research.

## Figures and Tables

**Figure 1:** The expression of nestin mRNA in the myeloid leukemia group and control group.

**Figure 2:** The expression of Keap1, Nrf2, and HO-1 mRNA in the myeloid leukemia group and control group.

**Table 1:** General patient information.

Groups	Control group	Leukemia group
Sex (M/F)	10/10	12/8
Age	36.75 ± 4.69	38.21 ± 5.17
Leukocyte count	5.89 × 10^3^	1.36 × 10^9^

## Data Availability

No data were used to support this study.
